The article "Predicting the Growth of F. proliferatum and F. culmorum and the Growth of Mycotoxin Using Machine Learning Approach" was retracted in 2023. Reasons: signs of a paper mill; suspected computer-generated content; unreliable results or conclusions; concerns about the data.

# Predicting the Growth of F. proliferatum and F. culmorum and the Growth of Mycotoxin Using Machine Learning Approach

**DOI:** 10.1155/2022/9592365

**Published:** 2022-07-15

**Authors:** R. Srinivasan, T. Lalitha, N. C. Brintha, T. N. Sterlin Minish, Sami Al Obaid, Sulaiman Ali Alharbi, S. R. Sundaram, Jenifer Mahilraj

**Affiliations:** ^1^Department of Computer Science and Engineering, Vel Tech Rangarajan Dr. Sagunthala R&D Institute of Science and Technology, Avadi, 600054 Tamil Nadu, India; ^2^Department of Computer Science and Engineering, VIT University, Chennai, 632014 Tamil Nadu, India; ^3^Department of Computer Science and Engineering, Kalasalingam Academy of Research and Education, Anandnagar, Krishnankoil, 626126 Tamil Nadu, India; ^4^Department of Computer Science and Engineering, Presidency University, Bengaluru, Yelahanka, 560064 Karnataka, India; ^5^Department of Botany and Microbiology, College of Science, King Saud University, PO Box 2455, Riyadh 11451, Saudi Arabia; ^6^Department of Sciences, University of Tennessee Health Science Center, Memphis, TN 38103, USA; ^7^Department of CSE & IT, School of Engineering and Technology, Kebridehar University, Ethiopia

## Abstract

In distinct parts of the food web, Fusarium culmorum and Fusarium preserving the relationship can germinate and grow zearalenone (ZEA) and fumonisins (FUM), accordingly. Antimicrobial drugs used to combat these fungi and toxic metabolites raise the risk of hazardous residue in food products, as well as the development of fungus tolerance. For modeling fungal growth and pathogenicity under separate water action (*a*_*q*_) (0.96 and 0.99) and surface temp (20 and 28°C) tyrannies, several machine learning (ML) methodologies (artificial neural, regression trees, and extreme rise enhanced trees) and multiple regression model (MLR) were used also especially in comparison. GR and mycotoxin levels inside the environment often reduced as EOC concentrations grew, although some treatment in association with specific *a*_*q*_ and temperature values caused ZEA production. In terms of predicting the growth rate of F. culmorum and F. maintaining the relationship and the production of ZEA and FUM, random forest techniques outperformed neural network models and extreme gradient boosted trees. The MLR option was the most inefficient. It is the first research to look at the ML potential of bio EVOH products containing EOCs and ambient variables of F. culmorum and F. proliferatum development, as well as the generation of zearalenone and fumonisins. The findings show that these entire novel wrapping technologies, in tandem using machine learning techniques, could be useful in predicting and controlling the dangers connected with fungal species or biotoxins in foodstuff.

The article "Predicting the Growth of F. proliferatum and F. culmorum and the Growth of Mycotoxin Using Machine Learning Approach" was retracted in 2023. Reasons: signs of a paper mill; suspected computer-generated content; unreliable results or conclusions; concerns about the data.

## 1. Introduction

Fusarium proliferatum and Fusarium culmorum were binary prevalent phytopathogenic organisms that harm nourishment globally before, during, and after harvest. Fusarium culmorum is a kind of Fusarium. Saccardo is a major producer of zearalenone (ZEA), a hormonally chemical that binds to the oestrogen receptor and damages sperm cell and testicles tissue. This species can be located in a range of foods, including grains and soybeans. One of the principals fumonisin- (FUM-) producing species is F. proliferatum (Matsushima) Nirenberg [1]. FUMs are toxins linked to equestrian leukoencephalomalacia, rodent hepatic and renal cytotoxicity, pig pulmonary edoema, humanoid esophageal tumor, and neural tube abnormalities. The International Agency for Research on Cancer has designated FUM, particularly fumonisin B1 (FB1), as potentially carcinogenic to humans (Group 2B). F. proliferatum can be originated in a variety of foods, including grains, soybeans, date palm plants, and tomatoes. As a result, FUM and ZEA, particularly FB1 and fumonisin B2 (FB2), are substances found in food across the globe. According to the United Nations Food and Agriculture, despite any use of chemical antimicrobial drugs for a prolonged time to monitor bacterial growth and mycotoxin generation in food, over 100 million metric tonnes of nourishment is ruined globally every year because of contamination caused by storing moulds [2]. Consumer preferences for fewer chemical additions to limit microbial development in foods while retaining quality, authenticity, and security exacerbate the situation. As a result, new methods are being created. Bioactive effective antibacterial technologies are a viable choice and an interesting way for improving the safety and quality of food in this sector. In the so-called barrier technique, it is an innovation that may be used in conjunction with each other.

Fusarium is one of the most notable fungi in nutritional mycology. Fusarium is a large species of fiber fungus that is part of a group often referred to as hypomycetes, which are widely distributed in the soil and associated with plants. Contamination with Fusarium spp. causes a decline in crop quality and productivity. Moreover, many of these species are capable of producing toxic secondary metabolites that can have adverse health effects on humans and animals [3]. Fusarium sporotrichioides and Fusarium langsethiae are the local Fusarium type of grains [4]. Both species are strongly linked and have a similar secondary metabolite spectrum. Both are found to create a large quantity of type A trichothecenes, such as HT-2 and T-2 toxins. Trichothecenes are harmful primarily because of their capacity to block protein synthesis and, at higher levels, operate primarily on actively dividing tissues such as marrow, lymph nodes, bone thymus, and intestinal mucosa. T-2 exhibits imprecise systemic effects, such as losing induces and weight organ failure, neurotoxicity, autoimmunity, haematotoxicity, and genotoxicity. T-2 is absorbed rapidly into a range of chemicals; it is most significant of which is HT-2. The toxin has been found in a variety of grain and cereal commodities, both commercially and organically grown barley, oats, wheat, and maize, according to multiple authors. Oats are the cereals with the greatest amount of both pollutants in general, notably in Central and Northern European countries [5]. F. langsethiae is the organism that causes this health concern in these countries. Antifungal therapies, as well as physicochemical factors (primarily water activity (aq)/comparative humidity and heat) which affect F. langsethiae development and T-2 and HT-2 generation, have been documented. Limited information is known about F. sporotrichioides' physicochemical needs, which could explain its geographical dispersion, a complicated issue that is currently unknown.

The article "Predicting the Growth of F. proliferatum and F. culmorum and the Growth of Mycotoxin Using Machine Learning Approach" was retracted in 2023. Reasons: signs of a paper mill; suspected computer-generated content; unreliable results or conclusions; concerns about the data.

Machine learning (ML) is a type of data framework that involves machines to understand from data and detect trends and regularities which are too complex for the human mind to recognise [6]. Machine learning is used to evaluate huge data sets and find patterns in the data that are linked to actual or perceived results. Many fields, such as probability and statistics, mathematics, and approximations concepts, are used in ML approaches. They can either be mostly monitored or completely unsupervised. In supervised machine learning, the input data is labelled based on a known outcome that the researchers are interested in. In supervised machine learning, a human sorts each data point in a training dataset, which includes both characteristics and outcomes. The purpose of supervised machine learning is to develop the optimal model for relating data and information [7]. A picture of a Petri dish with fermentation media, for illustration, could be categorized as “evolution extant” or “evolution missing.” A computer creates an algorithm to categorize each visual and compared its efficiency to the predefined “truth”; in most cases, initial results are insufficient; therefore, the system will continuously alter its settings by experimentation to boost performance.

A validation data is utilized to construct the final concept in this procedure. The evaluation can be done in a variety of ways. During the training phase, certain data is buried in these algorithms. Underfitting and overfitting are two issues that should be addressed throughout model construction. The technique based on the cross validation of *K*-fold for the training set is divided into *k* (typically 10) subgroups and is among the best ways to prevent the fitting problem [8]. Then, *k* times, a holdout learning approach is performed, with one of the *k* subsets serving as the validation dataset and the other *k* − 1 subsets serving as the training dataset. The training subset's measured variables are used throughout the validation process, so each opinion is being used only once for verification. The RMSE is an example of an error estimate measure that is average across all 10 trials [9]. Bias and variance are reduced as a result. A test set that was not seen in the training stage is often utilized to examine the ensuing model's generalization. Identification and prediction analysis can both benefit from supervised machine learning. Multiple regression (linear or logistic) and statistics categorization are the two most common supervised training techniques.

The article "Predicting the Growth of F. proliferatum and F. culmorum and the Growth of Mycotoxin Using Machine Learning Approach" was retracted in 2023. Reasons: signs of a paper mill; suspected computer-generated content; unreliable results or conclusions; concerns about the data.

Indispensable lubricants and their significant bioactive complexes, that are included in the generally regarded as safe (GRAS) classification, have been thoroughly researched as compared to the synthetic toxic substances in recent times, and various EO preparations are currently being analyzed and then used as natural preservatives [10]. Upwards of 17,000 aromatic flowering plants, mostly from the angiosperm groups Officinalis, Myrtaceae, Rutaceae, Brassicaceae, and Cyperaceae generate EOs. EO compositions can be immediately added to the mix or released slowly from product packaging. One of them is disinfection, which has minimal to no residual effects and is one of the best methods for preventing microbial infection throughout storage. When EOs are added to meals, bacteria populations are immediately reduced. The healing of wounded cells or the proliferation of cubicles that were not damaged by straight attachment may not have been stopped if the EO deposits are quickly exhausted due to its solubility [11]. Antimicrobial wrapping is a method that prevents or slows the growth of bacteria in food, hence extending the company's shelf life. Thus, the use of antibacterial products containing EOs allows the antibacterial to migrate to the coated surface and give a persistent antibacterial impact on the nourishment throughout time.

The environmental and organizational parameters used during various microbiological operations have a significant impact on the growth of a certain microbe. Modelling microbial development as an alternative to established microbiological procedures is gaining popularity. The framework that can forecast the growth of microbes and their comeback to various functioning circumstances must be developed and validated [12]. Because of its broad array of claims and ease with which it can grip deafening and extremely complicated data, ANN has gotten a lot of attention. The human brain can then be used to anticipate new input conditions after it has been trained. This is especially true in microorganism research findings, where microorganisms use biological neurocognitive processes to sense and respond to a range of data sources such as temperature, pH, agitation, and the appearance of energy metabolism components to achieve their existential objectives of survival, economic expansion, and reproductive capacity. Bacteria, like all living beings, respond to changing environments by altering their behaviours and metabolic.

The article "Predicting the Growth of F. proliferatum and F. culmorum and the Growth of Mycotoxin Using Machine Learning Approach" was retracted in 2023. Reasons: signs of a paper mill; suspected computer-generated content; unreliable results or conclusions; concerns about the data.

Essential oils (EOs) are the topic of multiple studies as a significant basis of sustainable and environment functional ingredients with good health advantages, as the need for “natural” antibacterial drugs has increased in last years, as nutrition safety gotten increased courtesy. Plant EOs' biological activity and preservation potential in food systems have been proven, leading to the conclusion that they could be a viable alternative to synthetic additives. The status of EOs has been upgraded to “commonly predicted as safe.” The US Food and Drug Administration (FDA) has accepted various flower EOs besides their constituents as additives, and the European Union (EC) has allowed them as well. Several essential oils include clove, thyme, eugenol, citral, cinnamaldehyde, carvone, and linalool. EOs must be enclosed in an appropriate delivery method for functional foods to sustain their bioactivity, decrease mobility, and raise effective usage amount, as well as minimize the negative impacts of their odor [13]. The most often investigated approach is directly mixing into container substrates. Smart packaging (SP) is a type of packaging that alters the circumstances of packaged meals to improve sensory or safety qualities and increase shelf life by shielding food from environmental and organizational influences when ensuring accuracy. This can be accomplished through the intrinsic features of the polymers utilized to make leather stuff or by adding dynamic ingredients to the initial vigorous packing or in the manufacturing process.

Ethylene-vinyl alcohol copolymers are polyester used in a variety of industries, including SP. The polymerization proportion of ethylene to vinyl alcohol determines the characteristics of EVOH. When compared to certain other polymers, copolymers with small ethylene concentration (below 33 mol percent ethylene) show superior block characteristics to *o*_2_ and smell under dry environments [14]. EVOH copolymers also have a high degree of transparency and remarkable mechanical characteristics. EVOH enriched with EOs or the unpolluted mechanisms have recently been shown to limit the growth of toxigenic fungus and mycotoxin generation. Active packaging material headspace of the SP can be regarded plastic films coupled with EOs. Antimicrobial packing is a kind of SP which not only protects but also outspreads the life of the product. In recent years, the use of these technologies in health sciences, such as microbiology, has exploded [15]. However, there has been little use of the machine learning field of analytical mycology, particularly the detection of fungal growth. Neural networks, including multilayer convolution layers and circular systems, are used to forecast fungal growth in food, as well as ochratoxin A making by Aspergillus carbonarius and deoxynivalenol manufacturing by Fusarium culmorum. Radio frequency is a nonlinear regression technique that is made out of ensembles of decision trees. They have been used to make predictions in mycology. Previous mycological studies have also found XGBoost to be beneficial. The goals of this interdisciplinary study were as follows: (1) analyze the effectiveness of EVOH integrating isoeugenol (IEG), citral (CIT), cinnamaldehyde (CINHO), or linalool (LIN) on the regulation of F. sporotrichioides expansion and the output of T-2 and HT-2 in oat cereals in various heat activity (*a*_*q*_) monarchies along the ultimate goal of discovering its applicability [16].

The article "Predicting the Growth of F. proliferatum and F. culmorum and the Growth of Mycotoxin Using Machine Learning Approach" was retracted in 2023. Reasons: signs of a paper mill; suspected computer-generated content; unreliable results or conclusions; concerns about the data.

Temperatures, water content (*a*_*q*_)/relative humidity (RH), and various antifungal medications all influence the development of pathogenic fungus like culmorum and proliferatum, as well as mycotoxin synthesis. These considerations have also been taken into account in research on the usefulness of bioactive films in preventing fungal proper growth and development of mycotoxin [6]. Many fields are involved in machine learning (ML) methodologies, including probability and statistics, economics, and approximations concept, and supervision ML can be utilized in hypothesis testing. Predictive model machine learning-based approaches can be useful tools for managing toxigenic fungus and mycotoxin generation, as well as for determining preventive therapies [3]. Neural network (NN) was used to forecast fungal infections or mycotoxin production by fungus, among other ML algorithms. Random forests (RF) are decision tree groups. They are supervised machine learning systems that have also been used to predict mycology. In a recent mycological investigation, excessive contributions to enhancing trees (XGBoost) were used.

The article "Predicting the Growth of F. proliferatum and F. culmorum and the Growth of Mycotoxin Using Machine Learning Approach" was retracted in 2023. Reasons: signs of a paper mill; suspected computer-generated content; unreliable results or conclusions; concerns about the data.

## 2. Related Work

Fusarium is fungus genera that comprise several forms that are harmful to grain and other products. Certain Fusarium species could create toxins that are harmful to both living creatures. Utilizing high-performance chromatography, zearalenone, fumonisin B2 and B1, trichothecenes kind A (toxin), and trichothecenes category B was investigated. Deoxynivalenol and zearalenone were discovered at quantities under European Union limitations in 72 percent and 38 percent of the grain specimens, correspondingly. Utilizing lifeform polymerase chain reaction techniques, the results are then compared to the existence of mycotoxigenic organisms thought to be responsible for the production. The existence of Fusarium verticillioides and fumonisin contamination and also zearalenone and F. graminearum presence, nivalenol, and deoxynivalenol residues in grain specimens were found to be quite reliable using genus polymerase chain reaction tests. F. sporotrichioides, F. culmorum, and F. poae, on the other hand, also were not found in some of the collections. The prevalence of the most major Fusarium toxicity in grain seedlings collected following European Union criteria was identified [17].

Herbs are supplied in developed economies having tropical and/or subtropical climates all around the globe. Extreme temperatures, torrential rains, and humidity encourage fungal infections, resulting in a rise in the presence of mycotoxins in spices. The report examines 38 different spices, 17 different mycotoxins, and 14 different microfungi. Spices are frequently disregarded in mycotoxin restrictions, which typically only apply to aflatoxins (AFs) and ochratoxin A. (OTA). The restrictions on mycotoxins in spices are discussed extensively in this study, both in the setting of the European Union (EU) and other territories. As the review has shown, the occurrence of AFs and OTA, as well as many other mycotoxins, is considerably large in numerous spices, necessitating the development of new regulatory limitations. Chili, nutmeg, and paprika powder have been the most problematic spices in terms of violating maximal EU restrictions, according to EU RASFF data. Such finding is backed up by data from individual research that were used to compile the analysis. Several other spices, nevertheless, were shown to contain AFs and OTA, as well as other mycotoxins in pretty substantial concentrations. The study compiles information comprising 56 original published papers during the past five years that focus on mycotoxins and microfungi in diverse spices [18].

The article "Predicting the Growth of F. proliferatum and F. culmorum and the Growth of Mycotoxin Using Machine Learning Approach" was retracted in 2023. Reasons: signs of a paper mill; suspected computer-generated content; unreliable results or conclusions; concerns about the data.

Acetone, ethanol, and methanol have been used to separate gilaburu. F. graminearum, F. oxysporum, F. coeruleum, F. sambucinum, F. solani, F. auneaceum, F. sulphureum, and F. culmorum are among Fusarium genotypes discovered. Overall, ethanolic extracts were shown to have the most antibacterial efficacy. Machine learning (ML) approaches were used to assess the antimicrobial activities of compounds. Many machine learning (ML) methodologies were used to predict fungal growth, including support vector machines (SVM), classification and regression trees (CART), artificial neural network (ANN), AdaBoost (AB) algorithm, ensemble algorithms (EA), random forests (RF), k-nearest neighbours bagging algorithm, and gradient boosting (GBM) algorithm as well as extra trees (ET). It is obvious from such a study that ML approaches have enough least mistake rates. As a consequence, machine learning techniques for estimating the antimicrobial activities of gilaburu isolates are efficient, quick, and inexpensive. These optimistic findings should encourage greater investigation into applying machine learning to the area of food microbiology rather than conventional methods. The work addresses the development of a numerical method to determine the thickness of the spontaneity area of gilaburu (Viburnum opulus L.) extract towards 8 several Fusarium isolates obtained in damaged potato tubers [19].

The Fusarium genus of infections is responsible for many of the world's most serious crop diseases. Almost all Fusarium species produce hazardous secondary metabolites classified as mycotoxins, although their functions are still unknown. Understanding that a fungal companion adapts its existence to fit in with the plant host is still a work in progress. It also focused on the metabolic processes and cytogenetic alterations which are impacted by mycotoxin interactions in plants. Furthermore, researchers investigated the synthesis of certain metabolites and mycotoxins in certain important fungal pathogen-plant host systems. Preventing Fusarium mycotoxins through plant techniques was also considered. Lastly, researchers reviewed the research on the role of plant subordinate metabolites in Fusarium disease defence. Considering multiple ecological variables, including moisture content, pH, temperature, and nitrogen source, the processes of mycotoxin production in the Fusarium species are given [8].

Fusarium head rot of grains has emerged as among the most serious preharvest illnesses in past years. Researchers are looking at how well fungicides work in the environment and in vitro to control Fusarium species in grains and the Fusarium illness of developing ears and its implications on mycotoxin production. According to field experiments, fungicides like tebuconazole and metconazole are effective at controlling both Fusarium disease of the ears and deoxynivalenol (DON) synthesis. Azoxystrobin and similar fungicides, on the other hand, are much less efficient, and grains of treated crops have occasionally been shown to have higher levels of DON and nivalenol. In research of Fusarium culmorum samples across various regions of Europe, complicated relationships among environmental conditions, fungicide variety, and isolation concerning inhibitory activity and DON generation were discovered. Such findings support azoxystrobin's incompetency and demonstrate that ecological stressors, such as water resources and temperatures, as well as low fungicide dosages, might accelerate Fusarium mycotoxin synthesis nonvitro and in cereal grains. The effectiveness of antimicrobials in suppressing Fusarium organisms in cereals in vitro and also their environmental efficiency on Fusarium infection of maturing earholes and their influence on toxin generation are examine [15].

The article "Predicting the Growth of F. proliferatum and F. culmorum and the Growth of Mycotoxin Using Machine Learning Approach" was retracted in 2023. Reasons: signs of a paper mill; suspected computer-generated content; unreliable results or conclusions; concerns about the data.

The requirement to maintain agricultural supply microbiology health and reliability has increased attention in statistical equations for measuring and forecasting microbial activities. To present, minimal advances have been made in the dynamical simulation of mycotoxins. Probabilistic algorithms could be an extra feature for predicting the likelihood of mycotoxin occurrence. Predicting a specific mycotoxin level, like the prescribed maximum, can be challenging since mycotoxin quantities are generally a result of the infecting fungus strain, except for ecological factors that may be used in modeling. Predicted microbiology was already created for the past 20 years to anticipate the frequency of food-borne diseases; likewise, such technologies are focused on microorganisms. The condition has somewhat changed, and a rising volume of investigations concerned only with prediction simulation methods of fungus are now accessible. The systematic study is about to the understanding to concentrate on predicting mycology and food security, involving mycotoxins; established kinetic and probability methods applicable to mycotoxigenic fungal yield and early, as well as mycotoxin production, are examined [18].

## 3. Materials and Methods

### 3.1. Film Preparation

The MELFIL Synthetic Chemical Industry Co., Ltd. provided an ethylene-vinyl alcohol copolymer (EVOH-29) with the molar concentration of 29 percent ethylene (Osaka, Japan). Sigma-Aldrich provided the linalool (LIN), trans-cinnamaldehyde (CINHO), isoeugenol (IEG), and citral (CIT) (Barcelona, Spain). Mateo et al. discussed how the films were made (2017a). In a nutshell, EVOH films with an initial content of 1, 2, 5, and 10% EOC are made by a moulding in a 75°C oven at 180. Cerisuelo et al. described thermal separation chromatography as a method for determining the ultimate amount of EOC. By evaluating polypropylene and polyethylene specimens with known quantities of CINHO, IEG, CIT, and LIN, the gas chromatograph's response was validated [3]. The additional content was determined as a mass ratio of the compounds over the dry mass polymer. Low fade, translucent, and uninterrupted EVOH-29 films carrying pure constituents of essential oils (Eos) were produced in all cases. According to the EOC type, the final levels for LIN, IEG, CIT, or CINHO discovered in the films were 0.37 ± 0.07 percent, 0.74 ± 0.11 percent, 1.85 ± 0.35 percent, and 3.8 ± 0.7%, *w*/*w* of dry polymer, for the films made at 1, 2, 5, and 10%, correspondingly.  Figure 1 shows the prediction model of machine learning. The functional EVOH films have a relevant dimension of 1.80 ± 0.01 mg/cm^2^. The biofilms are given the names EVOH-LIN, EVOH-IEG, EVOH-CINHO, and EVOH-CIT.

The article "Predicting the Growth of F. proliferatum and F. culmorum and the Growth of Mycotoxin Using Machine Learning Approach" was retracted in 2023. Reasons: signs of a paper mill; suspected computer-generated content; unreliable results or conclusions; concerns about the data.

### 3.2. Chemical, Reagents, and Mycotoxin Standards

LC-MS quality pure acetonitrile and grade pure methanol (MeOH) for the global teaching framework (MeCN). Bio B.V. provided formic acid with a ULC-MS grade of 99%. Sigma-Aldrich in Steinheim provided 99% ammonium formate and anhydrous magnesium sulfate. Merck (99%) provided formic acid analytical grade (92-100%) and sodium chloride (±92%). Millipore supplied Ultrafree®-MC centrifugal filters (0.3 *μ*m). On a Milli-Q Plus device, water was filtered to (15 M*σ*). Many of the other compounds and solutions were of importance to research. Sterigmatocystin (STERIG), aflatoxins B1 (AFB1), G1 (AFG1), B2 (AFB2), and G2 (AFG2) were bought from Sigma-Aldrich as mycotoxin benchmarks. Chromadex (California) provided O-methyl sterigmatocystin (OMST).

### 3.3. Inoculum Preparation

The strains F. culmorum Fc019 and F. proliferatum Fp06 were initially derived from a Spain grain. The genotypes are kept in the Stock Culture of the Mycology and Mycotoxins Group. The isolates were cultured on maize extraction medium (MEM), which consisted of 3 percent *w*/*v* powdered maize kernels plus +4% *w*/*v* agar in clear water. MEM was autoclave sterilized at (129°C for 50 minutes) before being transferred to Petri dishes [20]. Each endophytic fungus was seeded on the centre of the plates with (5 *μ*L) of bacterial culture (1 × 10^6^ spores/mL) and maintained for 7 days at 28°C. These new cells' conidia were utilized to make inocula for future research. Before every experiment, a fungal preparation containing (1 × 10^6^ spores/mL) was counted in shell chamber, and its monitoring was employed, and the solution was made with sterile Milli-Q water that contains 0.005% TWEEN 50.

The article "Predicting the Growth of F. proliferatum and F. culmorum and the Growth of Mycotoxin Using Machine Learning Approach" was retracted in 2023. Reasons: signs of a paper mill; suspected computer-generated content; unreliable results or conclusions; concerns about the data.

### 3.4. Fungal Isolates and Inoculum Preparation

Bioactive EVOH-EOC segments are tested in slightly milled maize grains (25 g) (pieces of 1–4 mm). Finely milled maize was inserted in Erlenmeyer bottles and then autoclaved for 30 minutes at 141 degrees Celsius to achieve toxic levels of ZEA, FB_1_, and FB_2_. Simultaneously time, flasks carrying milled maize were run to evaluate the activity *a*_*q*_ values exclusively. Then, using particular curves, ground maize is modified to 0.98 or 0.94 *a*_*q*_ by the injecting sterile filtered water. The aw-values were determined using regulations of defined aw values and a Novasina RTD 502 apparatus. The agar medium was placed in sterile Petri dishes with a diameter of 10 cm. Then, using dual sticky cellophane, a spherical portion (8 cm diameter) of each functional EVOH film with final dosages of 333, 666, 1665, and 3330 g of every EOC was placed to the edge of the Petri dish cover. The result of the quantity of each EOC in a film by the specific weight by the surface of the film yielded the final dosages of EOC per portion of the film. Initial tests were performed to determine the acceptable composition of each EOC injected into EVOH films to create dose-response curves. All surfaces in the Petri dish, including those without EVOH-EOC sheets, are vertically 15 l. A fresh conidia solution (1.106 conidia/mL) was used in the Proliferometer for Gulmoram before being parafilm-sealed. To create a constant balance humidity level inside the chambers, 3 samples of infected Petri dishes containing the same therapy (*a*_*q*_ and kind of film) were contained in sealed plastic tubs containing beakers of glycerol–water combination meeting the same aw as that of the therapy. Therapies and control samples were cultured in the shade for 20 days at 15 and 30 degrees Celsius. All of the trials were three replicates and repeatedly.

### 3.5. Effect of the Behaviours on a Mycotoxin Construction

#### 3.5.1. Mycotoxin Purpose in Cultures of Milled Maize

Irrespective of the size of an isolated fungi after the gestation period (21 days), the whole of growth (surface plus bacterial biomass) (about 25 g) in standards and therapies was taken from test tubes and dried at 35°C unless an equilibrium was reached. They are again excellently pulverized, standardized, and tested for the ZEA (F. culmorum cultures) and FB_1_ and FB_2_ (F. proliferatum cultures) using Tarazona et al.'s methods. Mycotoxins were collected from a portion of milling culture (2-3 g) in a Falcon tube using 8 mL water/formic acid/acetonitrile (80 : 19 : 1 *v*/*v*/*v*) under an orbital shaker for 1 hour. 2 mL of sample was collected through (0.22 *μ*m) PTFE syringe filter after sedimentation (4362 g, 7 min). Before even being injected into the analytical apparatus, samples from cells were concentrated (1 : 2 *v*/*v*) in the same solution. When aflatoxin levels exceeded the calibration curves range, the samples were mixed and administered again using that different solvent [21]. Density calibration was used for calibration reasons. Pure quantities of ZEA, FB_1_, and FB_2_ were dissolved in acetonitrile: water (1.1 *v*/*v*) and then diluted with organic solvent acid (19 : 1 *v*/*v*) to generate a mycotoxin stock solution. Additional measures were made by adding varying volumes of ZEA, FB_1_ or FB_2_ sample solution to extract noninoculated milling maize as described above for cultured. Blanks had previously been tested and determined to have no measurable levels of the relevant mycotoxins. The same isolating solvent was used to dilute dilutions of screened blank samples (1.2 *v*/*v*). Under a discharge of *N*_2_, aliquots of 2 mL of the concentrated extract were dried at room temperature, and suitable quantities of the standard were injected. For FB_1_ and FB_2_, the standardization range was 0.15–6.0 g/mL in the concentrated extract, while for ZEA, it was 0.055–5.0 g/mL. The areas of spots linked with the signifier ion of every component vs. mycotoxin level were calculated using scaled linear regression (weighted sum factor 1/*x*). Restoration assays and repetition of analyses were used to confirm the approach in-house, with some changes to mycotoxin doses and spiking intensities in restoration. In spiked blanks, mycotoxin values range from 2.65 to 250 g/g for ZEA, 50–160 g/g for FB_1_, and 3–50 g/g for FB_2_.

The article "Predicting the Growth of F. proliferatum and F. culmorum and the Growth of Mycotoxin Using Machine Learning Approach" was retracted in 2023. Reasons: signs of a paper mill; suspected computer-generated content; unreliable results or conclusions; concerns about the data.

#### 3.5.2. Effect of Treatments on Fungal Growth

Each day throughout the initial infection, the development of the experimental and reference cultures was measured and estimated by defining two sizes of the growing populations at sharp angles with a magnification [22]. The circumference of the colonies was calculated by multiplying both dimensions by four. File slopes are a collection by lagging analysis of the average population radius, the variation used to determine the circumference GR (mm/day). When applicable, the dosages of EOC in a EVOH film/plate required for 50%, 90%, and 100% growth arrest (AB_50_, AB_90_, and AB_100_) (the preceding AB is also referred as a minimum inhibitory concentration (MIC)) were calculated from GR vs. EVOH-EOC dose graphs. Several tests are successfully achieved and tested again.

#### 3.5.3. UPLC-MS/MS Conditions

The UPLC–MS/MS system comprised of an ACQUITY UPLC^TM^ equipment with a protonated mode (ESI+) access to these service ionization interfaces (ESI). The isolation was done in an ACQUITY UPLC BEH C18  column (50 × 2.1 mm and 1.7 m grain size) at 25°C. At a fluid velocity of 0.37 mL/min, the working fluid was a thing mixture of water comprising ammonium formate (0.15 mol/L) and the formic acid (0.1 percent) (solvent A) and methanol (solvent B) [23]. A total of 30 liters of fluid were injected. An ACQUITY TQD tandem quadrupole frame spectrometer was used to perform MS/MS detection. For every mycotoxin, two productions were measured. Data was collected using the Masslynx 4.2^TM^ chromatographic program and processed. An ACQUITY UPLC^TM^ a system with an electro-deposition was used in the UPLC–MS system. The diagnosis was based on the residence time of the targeted features in multireaction monitoring (MRM) analysis results.

#### 3.5.4. F. Sporotrichosis' Prediction Using a Machine Learning Algorithm

Upon that training sample, which has been selected randomly as from the entire dataset, the NN, SVM, XGBoost, and RF algorithms were developed and verified utilizing 10-fold cross-validation. The process framework is depicted in Figure 2 as a diagram.  Figure 3 depicts the dataset dynamically.

Supplementary shows the variance in root mean square error (RMSE) for different machine learning algorithms during strength and conditioning stages for prediction GR. Additional shows the RMSE difference for T-2 and HT-2 using different techniques. The least-square approach was used to predict the parameters of MLR solutions, and the data utilized for this operation was the same as that used only for learning and verifying the other algorithms. This regression analysis method begins with the set of data points projected on the *x*- and *y*-axis graph. An analyst who uses the minimum squares method will create a sequence of optimal matches that illustrate the possible relationship between independent and dependent variables [24].  Table 1 lists the features of the strongest ML representations discovered, as well as their RMSE and *R*^2^ values when matched to the test sample. For each output variable, five hypotheses were evaluated on the very same data set. The training dataset will not be used for learning or least square method adjustment (MLR).  Table 1 third column contains the optimal parameters for every ML model.  Figure 3 shows the graph for the performance of GR, T-2, and HT-2.

To acquire the best results, RF is always utilized a greatest number of specific response variables (mtry = 4), and SVM always utilized the similar rate for the regularisation limitation (*C* = 1) to have the greatest results. Whenever the RMSE (the chosen metrics) hits a low value, as well as the *R*^2^ value, approaches the unit, modeling performance is improved. The models with the smallest RMSE values typically had the highest *R*^2^ values as in Table 1.

The article "Predicting the Growth of F. proliferatum and F. culmorum and the Growth of Mycotoxin Using Machine Learning Approach" was retracted in 2023. Reasons: signs of a paper mill; suspected computer-generated content; unreliable results or conclusions; concerns about the data.

Additional Figure 3(a) shows the frequency distributions along with the lines of predicted standards for all the generated ML representations upon that test datasets for the GR and additional Figure 3(b) and additional Figure 3(c) for T-2 and HT-2, correspondingly. The *X*-score is a measured output charge for each location on the graphical representations. The *Y*-score of blue dots is the model's anticipated output variable; the *Y*-score of spots here on the fitted line is the figure's ideal expected estimated value if *Y* and *X* had a linear connection. The particles are also the distinction between the various *Y* coordinate values [25]. *Y* = *X* (slope = 1, intercept = 0) is the optimum line of perfect match, with no posterior probability and consequently RMSE = 0 and *R*^2^ = 1. In the testing dataset, the paths of the right candidate for XGBoost and NN to model GR statistically significant match (*p* value = 0.05) the paths of a perfect replacement, so the first had much less remaining variability, and the beginning reaches zero more. For trying to predict HT-2 toxin in a test dataset, it also tends to happen with XGBoost and RF. The gradient of the XGBoost figure's best-fitting line was numerically the unit for T-2, but still, the intersection was not negative.

## 4. Data Analysis

### 4.1. Analysis of Variance

The results were recorded using the Statgraphics Centurion XVII statistical software and multivariate regression analysis of variance (ANOVA). When ANOVA showed significant differences from among levels, post hoc Tukey's honestly significant difference was commonly employed to find homogeneous groups. To minimize spreading, the GR and saturation values were processed along (*x* + 1), where *x* was the raw quantity of the parameter.

### 4.2. Machine Learning Development

The machine learning approaches for simulating fungal GR and mycotoxin generation in cultures that were compared were XGBoost with RF (randomForest library) and NN (neuralnet library) (XGBTree library). The technique that was used was previously stated. A multiple linear regression (MLR) model was created for each reliant target value for fair comparison (outcome). The general form of the equation is

(1) $$\begin{array}{c} X=\delta_{0+}\overset{n}{\underset{m=1}{\sum }}\delta_{1}x_{1}+\mu \left(m=1,2,\cdots \cdots n\right), \end{array}$$

where *X* represents the output, *δ*_*o*_ is an independent variable, *δ*_1_*x*_1_ are the estimated coefficients, and these are predictors, *R*, and the “classifier training” (caret) module was used. Similar treatments were given to the two organisms. Heat, *a*_*q*_, type of EOC, and the EOC percentage were the four different variables. The secondary outcomes were (i) F. proliferatum, (ii) construction of FB2 by F. proliferatum, (iii) GR of F. culmorum, (iv) making of FB1 by F. proliferatum, and (v) construction of ZEA by F. culmorum. To mitigate risks, the results obtained were calculated based on datasets. Variables were preprocessed in some way. To prevent issues with unnoticeable concentration levels, the proportion of mean mycotoxin concentration plus 1 was calculated for mycotoxin results. Categorized data is recompiled as a set of classified data. Statistics set *R* performed mechanical rewriting (pseudo-coding). To avoid collinearity, *j* − 1 latent variables were installed for statistics with layers [3]. The numerical scales are not presented; the values of all other values are assessed about the base value. Every set of data (75 per output) was randomized divided into a training (85%) and test (15%) sets for the machine learning models. The learning algorithm was utilized to create and authenticate the models, while the testing set was cast away to assess its presentation on unrelated external information that had not been exposed to the representations earlier [20]. The parameters are selected to minimalize the quantity of the squared of the regressions in MLR, which is a linear regression technique that does not need a moment process for optimization (least-square method). The median adjusted square (RMSE) for training across the 10-fold pass was used to assess the machine learning techniques' performance. Boring process is a resampling technique for evaluating machine learning models on a small data sample. In comparison to previous techniques, it produces a less prejudiced estimate of system skill. The data is separated into ten subgroups in 10-fold bridge. A holding approach is repeated ten times, with one of the ten subsets serving as the testing dataset and the other nine subsets forming the training set. As a result, all recorded values in the educate subgroup are used for either training or test, with each comment being used only once for verification [14]. Because most of the variables are used for matching and since most of the variables are used in the testing set, the error prediction (RMSE) is averaged over all ten trials that minimizes bias and variation. The machine learning representations were fine-tuned to optimize their efficiency for each task based on the most important factors as shown in Table 2. Each model's *R*^2^ (coefficient of determination) value was calculated and averaged across all ten-fold cross-validation runs. All prediction models were evaluated and associated to a testing data (35 percent of the total dataset) that was not utilised to train or pass the models. These sets' RMSE and *R*^2^ values were calculated.

The article "Predicting the Growth of F. proliferatum and F. culmorum and the Growth of Mycotoxin Using Machine Learning Approach" was retracted in 2023. Reasons: signs of a paper mill; suspected computer-generated content; unreliable results or conclusions; concerns about the data.

### 4.3. Flowchart and Algorithm

In Figure 4, five independent factors have been used as input factors to the ANN, with the nondimensional outcome variable as the goal. The hidden sheet gathers the data of every linked node and transmits that to the output nodes. The estimated absorption spectrum is used to demonstrate the remedy at the output nodes. The total amount of data obtainable is separated into two collections, training, and testing dataset *t*. The training data set is utilized to construct the prediction models, while the test dataset is utilized to assess the model's predicting capabilities. Seventy percent of the data that is generated will be used for the training process, while the remaining 30% would be used as a test set. There were 295 diversity situations created from a random combined effect of all input variables. After that, 70% of the cultivation conditions were randomly chosen for the training phase and development monitoring. For forecasting, a residual 30% of cultures were chosen [26]. The MLR approach, developed by French philosophers, is frequently utilized in biomedical sciences and several other fields in which the measurement items are not overly associated. RMSE is the square root of the average squared error in the estimated value, which measures the overall accuracy of the model and is the basis for comparison with other models. The quantitative metrics RMSE and *R*^2^ were used to assess the algorithms' forecasting power. The root mean square error (RMSE) is the most commonly used universal error statistics. It is the square root of the mean of the square's errors among expected and actual values. The RMSE has always been positive, and the rate of 0 implies that the fit is optimal. Because RMSE gives huge mistakes a heavy strength, this is most effective whenever large errors are desired. The percentage of variation in the regression model due to the independent factors is known as *R*^2^.

## 5. Result and Discussion

### 5.1. Antifungal Methods of Bioactive EVOH-EOC Films

When growth occurred, all of the bacterial cultures in this investigation had round, plainly visible, and measured colonies. According to the cultural conditions, there is 3 to 5 days lag in growth. Significant changes in radial GR were reported in the change in organization by not using any film or films without EOC, in the same situation F. Gulmoram and F. Proliferation is maintained in the radiated GR of the colonies and in the standard and treatments. Different conditions are assessed (temperature and aw). As a result, the values displayed for Fusarium culmorum and Fusarium proliferatum control cultures, respectively, represent the average of the six repetitions of each 3 replicates as shown in Figures 5 and 6.

The article "Predicting the Growth of F. proliferatum and F. culmorum and the Growth of Mycotoxin Using Machine Learning Approach" was retracted in 2023. Reasons: signs of a paper mill; suspected computer-generated content; unreliable results or conclusions; concerns about the data.

At 28°C, the two organisms grew quicker than at 20°C, and at 0.98 *α*_*w*_, they went higher than at 0.97 *α*_*w*_. The growth rate of Fusarium culmorum is considerably advanced than the GR of Fusarium proliferatum under the same conditions. As a result, their actions were examined individually. ANOVA revealed that the kinds of antimicrobial agent, EOC dosages, and temperature have a substantial impact on the GR of F. culmorum and F. proliferatum (*p* < 0.05). Aw had a considerable impact on the growth rate of Fusarium proliferatum. The antimicrobial agent dose and heat aw interactions (for F. culmorum) and the antimicrobial agent dose and antimicrobial agent heat aw contacts (for F. proliferatum) were both significant (*p* < 0.05). Because there are significantly different (*p* < 0.05), more than one category is present. The kind of two homogeneous groups in bioactive EVOH film and the efficiency is (EVOH-CIT>IVOH-IEG≅EVOH-CINHO≈EVOH-LIN).

Table 3 shows the film efficiency derived from the Tukey HSD test (EVOH-CIT>EVOH-CINHO>EVOH-IEG>EVOH-LIN). In general, the larger the dose, the more effective the inhibition of fungal development is for both fungi. The Tukey HSD test was used to classify the four doses into three homogeneous clusters (3250-1465, 1465-555, and 444 g/Petri plate). When it comes to Fusarium culmorum, independent of dose, the mycelium performed better in holding back than in EVOH-CIT therapies. The two massive levels of EVOH-IEG (3250-1465 g/Petri plate) considerably reduced GR when compared to controls. The impacts of EVOH-EOC film type, EOC dosage, heat, and water content of Fusarium culmorum and F. proliferatum growth rate on partially pulverized maize kernels were studied using a post hoc Tukey's HSD test (= 0.05).

Only the maximum dose in EVOH-LIN significantly reduced GR as compared with the control group. Tukey HSD test identified dosages and controls in a homogenous group using EVOH-CINHO. Except for the lowest effective dose (444 g/Petri dish), all doses significantly reduced GR in F. proliferatum cultures compared to controls. Depending on the level of EVOH-EOC film, fungi pathogens, aq, and heat, the EDs to decrease the fungi's GR by 40%, 80%, and 100% ED_40,_ED_80, _ED_100_ were 100 to >3220 and 350 to >3220 and 390 to >3220 g of EOC/fungal culture, accordingly. F. culmorum demonstrated the highest sensitivity to every active EVOH films at 25°C and 0.98 *a*_*w*_, with a few exclusions. However, the effect of climatic variables on Fusarium proliferatum susceptibility to EVOH-EOC films was unclear and varied depending on the film examined. So, the smallest EDs for EVOH-CIT films have been investigated at 28°C and 0.98 *a*_*w*_, while the least EDs for EVOH-CINHO films that are observed at 30°C and 0.94 *a*_*w*_.  Table 4 provides the effective dosage of EVOH-EOC film/Petri plate. Overall, the EVOH-CIT therapies had the lowest EDs while the EVOH-LIN therapies had the greatest EDs when considering both species and all heat combinations.

The article "Predicting the Growth of F. proliferatum and F. culmorum and the Growth of Mycotoxin Using Machine Learning Approach" was retracted in 2023. Reasons: signs of a paper mill; suspected computer-generated content; unreliable results or conclusions; concerns about the data.

The residuals higher testing set than training dataset, and the random forest algorithms had the finest (lowest) highest accuracy. In the case of FB2, however, similar root mean square numerals are estimated for the RF and gradient boosting models. The MLR models had the greatest root mean square error values and the least *R*^2^ for the test set. According to the conclusion, the comparative performance of NN and XGBoost was altered. The broken plots show you anticipated against actual results for the RF and MLR models applied to the identical test sets for Fusarium culmorum growth rate and F. proliferatum's production of ZEA FB_1_ and FB_2_, respectively. Disadvantage expected numbers found with MLR models are meaningless and were treated as zero. There are no guesstimates (predictions) out of the confines of the measured output values, which is a property of RF. RMSE values are only useful for comparing models on a specific outcome, not for comparing models in general. The computed outputs for toxins were mentioned in the following:

(2) $$\begin{array}{c} \left(\ln\left(C\right.\left(\text{ZEA}\right)+1\right),\ln\left(C\right.\left(\text{ZEA}\right)+1,\ln\left(C\left({\text{FB}}_{1}\right)+1\right)+\ln\left(C\left({\text{FB}}_{2}\right)+1\right), \end{array}$$

where ln represents natural logarithm and *C*(ZEA), *C*(FB_1_), and *C*(FB_2_), respectively, are concentrations of ZEA, FB_1_, and FB_2_.

## 6. Conclusion

Fusarium culmorum as well as Fusarium proliferatum grew faster at 28°C than at 20°C and at 0.99 aw than at 0.96 aw, as per our findings. The GR of F. second most widely was substantially larger than the GR of F. proliferatum together under the circumstances. *a*_*q*_, temperatures, and treatments all influenced fungal infections and ZEA and FUM generation. EVOH-CIT, EVOH-IEG, and EVOH-CINHO are postulated as the most potential candidate for therapeutic interventions against F. culmorum and F. proliferatum and as modulators of ZEA and FUM manufacturing, based on the effectiveness of the EVOH-EOC films assayed, as reflected by the ED points, suppression of microbial GR, stoppage of mycotoxin biosynthetic pathway, and the relative cost of the E. In comparison to the multiple linear regression, which had an *R*^2^ of 0.8, the ANN model was used to predict the distributed development efficiently. The findings support the use of the prediction over multiple linear regression in the development of methods to better forecast the distributed development of microorganisms. Several researches have found that using an experiment database, neural nets can predict the exact growth of microorganisms. Currently, lethal EOC dosages against toxigenic F. oxysporum are being implemented. As a pretty effective method of preventing fungal proliferation and the creation of mycotoxin in food, it could become problematic. The few researches have used machine learning to forecast the growth of toxigenic fungi and the generation of mycotoxin reveal. These techniques can be incredibly beneficial in preventing and managing these dangers. RF algorithms were able to accurately predict F.'s GR among some of the machine learning investigated in this research. F. culmorum and culmorum neural network, XGBoost, and multiple linear regression algorithms produced more mycotoxin as well as proliferatum (ZEA and FUM) than neural network, XGBoost, and multiple linear regression models.

The article "Predicting the Growth of F. proliferatum and F. culmorum and the Growth of Mycotoxin Using Machine Learning Approach" was retracted in 2023. Reasons: signs of a paper mill; suspected computer-generated content; unreliable results or conclusions; concerns about the data.

## Figures and Tables

**Figure 1:** A prediction model.

**Figure 2:** Machine learning algorithm framework.

**Figure 3:** Graph for the performance of GR, T-2, and HT-2.

**Figure 4:** Flowchart of methodology.

**Figure 5:** Radial GR of F. culmorum dosages, control measurements, and treatments.

**Figure 6:** Radial GR of F. proliferatum colony dosages, control measurements, and treatments.

**Algorithm 1:** Machine learning algorithm.

**Table 1:** Performance of ML models for predicting the growth rate, HR-2, and T-2.

Output parameter	Machine learning tested model	Parameter of best model	RMSE^*a*^	*R* ^2^*b*^^
Growth rate	XGBoost	Dimension = 5; decay = 0.4, ntree = 500, mtry = 4, max_depth = 7, eta = 0.1, *C* = 2, subsample = 1	1.445	0.866
	Artificial neural network		1.265	0.898
	SVM		1.162	0.921
	Random forest		1.542	0.918
	MLR		1.670	0.845
Production of T-2	XGBoost	Dimension = 5; decay = 0.2, ntree = 500, mtry = 4, max_depth = 2, eta = 0.1, *C* = 1, subsample = 1	0.768	0.795
	Artificial neural network		0.402	0.945
	SVM		0.356	0.765
	Random forest		0.623	0.787
	MLR		0.635	0.765
Production of HT-2	XGBoost	Dimension = 2; decay = 0.4, ntree = 500, mtry = 7, max_depth = 6, eta = 0.3, *C* = 1, subsample = 1	0.543	0.723
	Artificial neural network		0.525	0.782
	SVM		0.567	0.805
	Random forest		0.543	0.775
	MLR		0.885	0.764

The article "Predicting the Growth of F. proliferatum and F. culmorum and the Growth of Mycotoxin Using Machine Learning Approach" was retracted in 2023. Reasons: signs of a paper mill; suspected computer-generated content; unreliable results or conclusions; concerns about the data.

**Table 2:** Machine learning main parameter model and their values.

Machine learning model	Name of the parameter	Description	Standard values
Neural network	Decay	Decay rate weight	[0.2, 0.4, 0.6]
	Size	Unit of hidden layer	[5, 10, 15, 20, 25]
Random forest	ntree	Number of trees	500
	mtry	A randomly selected number of predictors	[2, 3, 5]
Extreme gradient boosted tree	Max_depth	Maximum of tree depth	[0, 1, 2, 3, 4, 5]
	Gamma	Penalty factor regularization	0
	nrounds	Number of iterations	150
	Colsample_bytree	Column fraction to be arbitrarily tested for every tree	1
	Subsample	Subsample percentage from the training established to cultivate a tree	[0.5, 0.75, 1, 1.25]
	Minimum_child_weight	Weight of low weight instance per node	0.5
	Eta	Shrinkage or rate of learning	[0.1, 0.2, 0.3]

**Table 3:** The film efficiency.

Regions	Level	Bacterial spices					
		F. culmorum		F. proliferatum			
		Rate of growth		Rate of growth			
		Low to high		Low to high			
EVOH-EOC films	CIT	^∗^		^∗^			
	IEG		^∗^		^∗^		
	CINHO		^∗^			^∗^	
	LIN		^∗^				^∗^
Dosage (*μ*g EOC/Petri dish)	444	^∗^				^∗^	
	555	^∗^			^∗^		
	1465	^∗^			^∗^		
	3250		^∗^		^∗^		
Heat (°C)	25	^∗^			^∗^		
	30	^∗^					
Activity of water	0.96		^∗^			^∗^	
	0.99						^∗^

**Table 4:** The effective dosage of EVOH-EOC film/Petri plate.

Spices	Heat °C	*∂*_*w*_	Ethylene vinyl-trans-cinnamaldehyde			Ethylene vinyl-citral			Ethylene vinyl-isoeugenol			Ethylene vinyl-linalool		
			ED_40_	ED_80_	ED_100_	ED_40_	ED_80_	ED_100_	ED_40_	ED_80_	ED_100_	ED_40_	ED_80_	ED_100_
F. culmorum	28	0.94	2300	>3080	>3080	437	436	560	1200	>3080	>3080	2450	>3080	>3080
		0.98	580	1332	1325	300	453	560	780	1332	1325	670	>3080	>3080
	30													
		0.94	470	765	3080	733	243	560	568	765	3080	540	>3080	>3080
F. proliferatum	28	0.98	3080	>3080	670	654	987	560	983	>3080	670	>3080	>3080	>3080
		0.94	>890	>896	670	984	548	560	780	>896	670	>3080	>3080	>3080
	30													
		0.98	>3080	>3080	3080	900	850	560	450	>3080	3080	>3080	>3080	>3080

## Data Availability

The data used to support the findings of this study are included within the article. Further data or information is available from the corresponding author upon request.
